# Fractional-Order Ebola-Malaria Coinfection Model with a Focus on Detection and Treatment Rate

**DOI:** 10.1155/2022/6502598

**Published:** 2022-09-16

**Authors:** Lingling Zhang, Emmanuel Addai, Joseph Ackora-Prah, Yarhands Dissou Arthur, Joshua Kiddy K. Asamoah

**Affiliations:** ^1^Department of Mathematics, Taiyuan University of Technology, Shanxi Taiyuan 030024, China; ^2^Department of Mathematics, Kwame Nkrumah University of Science and Technology, Kumasi, Ghana; ^3^Department of Mathematics Education, Akenten Appiah-Menka University of Skills Training and Entrepreneurial Development, Kumasi, Ghana

## Abstract

Coinfection of Ebola virus and malaria is widespread, particularly in impoverished areas where malaria is already ubiquitous. Epidemics of Ebola virus disease arise on a sporadic basis in African nations with a high malaria burden. An observational study discovered that patients in Sierra Leone's Ebola treatment centers were routinely infected with malaria parasites, increasing the risk of death. In this paper, we study Ebola-malaria coinfections under the generalized Mittag-Leffler kernel fractional derivative. The Banach fixed point theorem and the Krasnoselskii type are used to analyse the model's existence and uniqueness. We discuss the model stability using the Hyers-Ulam functional analysis. The numerical scheme for the Ebola-malaria coinfections using Lagrange interpolation is presented. The numerical trajectories show that the prevalence of Ebola-malaria coinfections ranged from low to moderate depending on memory. This means that controlling the disease requires adequate knowledge of the past history of the dynamics of both malaria and Ebola. The graphical dynamics of the detection rate indicate that a variation in the detection rate only affects the following compartments: individuals that are latently infected with the Ebola, Ebola virus afflicted people who went unnoticed, individuals who have been infected with the Ebola virus and have been diagnosed with the disease, and persons undergoing Ebola virus therapy.

## 1. Introduction

Malaria is a dangerous and occasionally deadly disease that can cause altered body posture, irregular eye movements, paralysis of eye movements, and coma. The World Health Organization estimates that millions of people worldwide have contracted malaria and thousands have died as a result of it, the majority of whom are youngsters in Africa. Commuters returning from places of the world where malaria transmission occurs, such as sub-Saharan Africa, make up the great majority of cases. Malaria is a potentially fatal disease, yet it is frequently preventable. According to estimates, malaria costs sub-Saharan Africa billion of dollars every year [1, 2]. Ebola virus disease outbreaks occur on a rare basis in African countries where malaria is already a major problem. The majority of Ebola virus disease outbreaks have been minor in the past, with case counts typically under 100 people [3].

Epidemiological modeling of infectious diseases using integer-order differential equations to explore and investigate epidemic transmission dynamics has been in existence for many years. The advancement of fractional calculus has revealed important information about disease transmission patterns or dynamical behaviors. In the study of biological and engineering systems, fractional order differential equations have proved themselves as powerful and effective mathematical modeling tools. This is because most often differential operators that are found in these equations or models are associated with memory dynamics, which can be seen in biological and engineering systems [4]. The Mittag-Leffler kernel derivative has recently been utilised to mimic a variety of real-world occurrences, for example [5, 6], using the three fractional derivatives, the authors of [7] analysed the dynamics of the Q fever epidemic. From their research, they deduced that, unlike the integer order, the trajectories of some fractional orders converge to the same endemic equilibrium point. In conclusion, it was found that the Atangana-Baleanu fractional differential operator captures more susceptibilities while allowing for a smaller number of infections. Existence-uniqueness, stability, and simulated solutions to the HIV/AIDS infection model were analysed using the Mittag-Leffler kernel by the authors of [8]. Okyere et al. [9] studied an SIR model using the Caputo derivative. Using the same operator, the work in [10] studied the dynamics of COVID-19 and presented the usefulness of memory in the transmission of COVID-19. Erturk et al. [11] presented a study to describe motion of beam on nanowire. As the order of the fraction increases toward unity, their findings show that the fractional responses become increasingly similar to the classical ones. The fractional Euler-Lagrange equation also provides a flexible model with more information than the classical description, which allows for a much more accurate assessment of the system's hidden features. Jajarmi et al. [12], applied fractional-order to study capacitor microphone. Results show that, in contrast to the previous mathematical formalism, the freedom to choose the kernel allows for the discovery of new properties of the capacitor microphone under investigation. Baleanu et al. [13] studied the relative importance of memory on cholera outbreak. The work in [14] presented some applications of a regularized Ψ-Hilfer fractional derivative.

The 2014 Ebola virus epidemic in three sub-Saharan African countries, namely Guinea, Liberia, and Sierra Leone, was considered to be significant, with approximately 28,616 suspected and confirmed cases and over 11,310 deaths in these three majorally affected countries in sub-Saharan Africa. To examine the spread of Ebola virus disease transmission in Sub-Saharan African countries, Berge et al. [15] developed a vulnerable infected-recovered-death model, with natural mortality in susceptible-infected-recovered (SIR) compartments, it was assumed that recovered individuals lost immunity and became susceptible again. Chowell and Nishiura [16] studied the transmission dynamics and control of Ebola virus disease. Omeloye and Adewale [17] presented a mathematical analysis on Ebola-malaria transmission dynamics, demonstrating that if the detection rate of infected undiscovered persons is high enough, isolation can lead to Ebola eradication in the population. Furthermore, Omeloye and Adewale [18] created an optimal control in the Ebola-malaria coinfection model. They studied the disease-free equilibrium of each model. Their co-infections were shown to be locally and globally asymptotically stable whenever the basic reproduction number is less than unity or endemic otherwise. Thus, prior mathematical investigation on Ebola-malaria coinfections has not taken into account the fractional derivative. As a result, our research add up to the dynamic analysis of Ebola, malaria, and Ebola-malaria coinfections. First and foremost, we guaranteed solutions of the existence and uniqueness by the use of the Krasnoselskii type and Banach fixed point theorem. And also, Hyers-Ulam stability guaranteed the model stability. Motivated by the work in [18] the current work contributes the following:

- A new fractional mathematical model for the co-dynamics of Ebola and malaria is considered and studied using the Atangana-Baleanu derivative [19]
- The existence and uniqueness of the solution of the proposed model employing the Banach fixed point theorem and the Krasnoselskii type are shown
- Using the generalized Mittag-Leffler kernel, we exhibited the rich dynamics of this disease when memory of past history of the disease is taken into consideration through simulations
- We highlight the impact of detection rate and treatment rate on the dynamics of coinfection of Ebola and malaria when the fractional order is 0.99, unlike the integer order of 1

The remainder of this paper is organized as follows: some critical concepts, basic definitions, and preliminary results are all briefly introduced in Section 2. In section 3 we restate the model formulation of the Ebola-malaria coinfection model and briefly describe all the parameters as in [18], and then impose the Mittag-Leffler kernel fractional derivative on the model.  Section 4 is devoted to the mathematical analysis of the existence-uniqueness of Ebola-malaria coinfection model. The stability results of the Ebola-malaria coinfections model are presented and discussed in Section 5. The numerical scheme and simulations are discussed in Section 6 and Section 7, respectively. The paper ends with a conclusion in Section 8.

## 2. Preliminaries

Now, we recall some critical ideas, lemmas, and definitions to study the system (11).

**Definition 1 (see [20, 21]).**

The ABC-fractional differential operator on Θ ∈ *H*^1^(*a*, *b*), for *ω* ∈ (0, 1) is

(1) D ABCσωΘσ=∇ω1−ω∫0σΘ′sEω−ωσ−sω1−ωds,

where ∇(*ω*) is the normalization constant that satisfies the property ∇(1) = ∇(0) = 1. And *E*_*ω*_ is the Mittag-Leffler function, which can be defined as

(2) $$\begin{array}{c} E_{\omega }\left(y\right)=\overset{\infty }{\underset{k=0}{\sum }}\frac{y^{k}}{\Gamma \left(\omega k+1\right)}. \end{array}$$

**Definition 2 (see [8]).**

For Θ ∈ *H*^1^(*a*, *b*) and for *ω* ∈ [0, 1], the ABC-fractional integral is given by;

(3) I ABCσωΘσ=1−ω∇ωΘσ+ω∇ωΓω∫0σΘsσ−sω−1ds,

assuming that the integral on the right converges.

**Lemma 1 (see [4]).**

From the ABC-fractional derivative and its integral of the function Θ, hold for the Newton-Leibniz formula:

(4) I ABCσωD ABCσωΘσ=Θσ−Θω.

**Lemma 2 (see [8]).**

Suppose that *y*(*σ*) ∈ *L*_*p*_[0, *η*], then the solution of fractional differential equation.

(5) D ABCσωΘσ=yσ,σ∈0,η,Θ0=Θ0,

is given by

(6) $$\begin{array}{c} \Theta \left(\sigma \right)=\Theta_{0}+\frac{1-\omega }{\nabla \left(\omega \right)}\Theta \left(\sigma \right)+\frac{\omega }{\nabla \left(\omega \right)\Gamma \left(\omega \right)}\int_{0}^{\sigma }\Theta \left(s\right){\left(\sigma -s\right)}^{\omega -1}ds. \end{array}$$

Now, we let *B* = *C*([0, 1]) be a Banach space with the following norm

(7) $$\begin{array}{c} \left\|\Theta \right\|=\underset{\sigma \in \left[0,\eta \right]}{\max}\left\{\left|\Theta \right|,\forall \Theta \in B\right\}. \end{array}$$

**Lemma 3 (see [22]).**

From the Krassnoselskii's fixed point theorem if we assume that *M* ⊂ *B*, be a closed convex non-empty subset of *B* and ∃ and two operators *Ω*_1_ and *Ω*_2_, then we will have the following:

- *Ω*_1_Θ + *Ω*_2_Θ ∈ *B*, ∀Θ ∈ *B*
- *Ω*_1_ is contraction and *Ω*_2_ is continuous and compact. Then there exist at least one solution Θ ∈ *B* such that

(8) $$\begin{array}{c} \Omega_{1}\Theta +\Omega_{2}\Theta =\Theta . \end{array}$$

## 3. Model Formulation

In this section, we formulate and explain the entire epidemiological compartments related to the human population and vector population at time *t*. The susceptible individuals is denoted by *S*_*H*_(*t*), *L*_*E*_(*t*) is individuals that are latently infected with the Ebola virus, *I*_*U*_(*t*) is Ebola virus afflicted people who went unnoticed, *I*_*D*_(*t*) is indicated as individuals who have been infected with the Ebola virus and have been diagnosed with the disease, *I*_*T*_(*t*) is persons undergoing Ebola virus therapy, *J*(*t*) denotes isolated Ebola individuals, malaria-exposed population is denoted as *E*_*M*_(*t*), *I*_*M*_(*t*) denotes malaria infected individuals, *R*_*M*_(*t*) represents people who have recovered from malaria, *E*_*EM*_(*t*) represents individuals who are infected with the Ebola virus and at the risk of contracting malaria, and *I*_*EM*_(*t*) denotes persons infected with Ebola and Malaria. The vector population is landmarked as follows: *S*_*V*_(*t*) represents susceptible to mosquitoes, *E*_*V*_(*t*) denotes exposed to mosquitoes, and *I*_*V*_(*t*) denotes infected with mosquitoes. *N*_*H*_(*t*) is the total human population and *N*_*V*_ is the total vector population. Considering the interrelationship with the compartments as referenced in [18] the following nonlinear ordinary differential equations represents the model formulation:

(9) $$\begin{array}{c} \left\{\begin{array}{c} \frac{dS_{H}}{dt}=\pi_{H}-\lambda_{E}S_{H}-\lambda_{M}S_{H}-\lambda_{EM}S_{H}-\mu S_{H}+\phi_{1}R_{M}+\alpha \theta J,\\ \frac{dL_{E}}{dt}=\varepsilon_{1}\lambda_{E}S_{H}-\left(K_{E}+\sigma_{1}+\mu \right)L_{E}+\phi_{2}I_{T}+\left(1-\alpha \right)\theta J-\left(1-\rho \right)\phi_{3}I_{EM},\\ \frac{dI_{U}}{dt}=\left(1-\varepsilon_{1}\right)\lambda_{E}S_{H}+\omega_{1}K_{E}L_{E}-\left(\gamma_{UE}+\mu +\delta_{UE}\right)I_{U},\\ \frac{dI_{D}}{dt}=\left(1-\omega_{1}\right)K_{E}L_{E}-\left(\tau_{1}+\mu +\delta_{ED}+\sigma_{2}\right)I_{D}+\gamma_{UE}I_{U}+\tau_{4}E_{EM},\\ \frac{dI_{T}}{dt}=\tau_{1}I_{D}-\left(\phi_{2}+\mu \right)I_{T},\\ \frac{dJ}{dt}=\sigma_{1}L_{E}+\sigma_{2}I_{D}-\left(\mu +\delta_{j}\right)J-\theta J,\\ \frac{dE_{M}}{dt}=\varepsilon_{2}\lambda_{M}S_{H}-\left(K_{M}+\mu \right)E_{M}-\tau_{2}E_{M}+\rho \phi_{3}I_{EM},\\ \frac{dI_{M}}{dt}=\left(1-\varepsilon_{2}\right)\lambda_{M}S_{H}+K_{M}E_{M}-\left(\tau_{3}+r+\delta_{IM}+\mu \right)I_{M},\\ \frac{dR_{M}}{dt}=\tau_{2}E_{M}+\tau_{3}I_{M}+rI_{M}-\left(\phi_{1}+\mu \right)R_{M},\\ \frac{dE_{EM}}{dt}=\varepsilon_{3}\lambda_{EM}S_{H}+\left(K_{EM}+\delta_{IEM}+\mu \right)E_{EM}-\tau_{4}E_{EM},\\ \frac{dI_{EM}}{dt}=\left(1-\varepsilon_{3}\right)\lambda_{EM}S_{H}+K_{EM}E_{EM}-\left(\phi_{3}+\delta_{IEM}+\mu \right)I_{EM},\\ \frac{dS_{V}}{dt}=\pi_{V}-\lambda_{V}S_{V}-\mu_{V}S_{V},\\ \frac{dE_{V}}{dt}=\lambda_{V}S_{V}-\left(\sigma_{V}+\mu_{V}\right)E_{V},\\ \frac{dI_{V}}{dt}=\sigma_{V}E_{V}-\mu_{V}I_{V}, \end{array}\right. \end{array}$$

where *λ*_*E*_, *λ*_*EM*_, *λ*_*M*_, and *λ*_*V*_ is defined as follows: *λ*_*E*_ = *β*_*E*_(*I*_*U*_ + *η*_*D*_*I*_*D*_ + *η*_*j*_*J*/*N*_*H*_), *λ*_*EM*_ = *β*_*EM*_(*E*_*EM*_ + *η*_*EM*_*I*_*EM*_/*N*_*H*_), *λ*_*V*_ = *β*_*V*_*b*(*I*_*M*_ + *η*_1_*E*_*EM*_ + *η*_2_*I*_*EM*_/*N*_*H*_), and *λ*_*M*_ = *β*_*M*_(*bI*_*V*_/*N*_*V*_).

The total population is given as;

(10) $$\begin{array}{c} N_{H}\left(t\right)=S_{H}\left(t\right)+L_{E}\left(t\right)+I_{U}\left(t\right)+I_{D}\left(t\right)+I_{T}\left(t\right)+J\left(t\right)+E_{M}\left(t\right)+I_{M}\left(t\right)+R_{M}\left(t\right)+E_{EM}\left(t\right)+I_{EM}\left(t\right), \end{array}$$

and *N*_*V*_(*t*) = *S*_*V*_(*t*) + *E*_*V*_(*t*) + *I*_*V*_(*t*).

The associated parameters considered in model (9) along with detailed descriptions are given as *π*_*H*_ and *π*_*V*_ are the recruitment rate of human and vectors, respectively, *λ*_*M*_ is the force of infection for malaria transmission, *λ*_*E*_ is the force of infection for the Ebola virus, *λ*_*EM*_ is the force of infection in *I*_*EM*_, *μ* is the human death rate, *μ*_*V*_ is the vector (mosquitoes) death rate, *τ*_1_ is the treatment rate for Ebola, *τ*_2_ is the malaria infected rate, *τ*_3_ denotes malaria treatment rate, *τ*_4_ is the exposed rate, and *ε*_1_ and *ε*_2_ are the Ebola and malaria low immunity rate, respectively. *ε*_3_ is the Ebola-malaria low immunity rate, *γ*_*UE*_ is the detection rate of unknown Ebola virus, *δ*_*EM*_ is the malaria induced death rate for *E*_*M*_, *δ*_*IM*_ is the malaria induced death rate for *I*_*M*_, *σ*_1_ and *σ*_2_ are the isolation rate for *L*_*H*_ and *I*_*D*_, respectively. *K*_*E*_, *K*_*M*_, and *K*_*EM*_ are the progression rate for malaria, Ebola, and Ebola-malaria, respectively, *δ*_*UE*_ and *δ*_*DE*_ are the Ebola induced death rate for *I*_*U*_.and *I*_*D*_, respectively, *δ*_*j*_, *δ*_*EM*_, and *δ*_*IEM*_ are the Ebola induced death rate for *J*, *E*_*EM*_, and *I*_*EM*_, respectively, *σ*_*V*_ is the progression rate vectors, and *ϕ*_1_ is the rate of loss of immunity. *β*_*E*_ and *β*_*EM*_ are the effective contact rate for Ebola virus and Ebola-malaria, *r* is the recovery rate of malaria, *λ*_*M*_ and *λ*_*V*_ are the force of infection from vector-human and human-mosquito, respectively, *ϕ*_3_ is the active rate of Ebola-malaria after treatment, *β*_*M*_ is the transmission rate from mosquito to human, *β*_*V*_ is the transmission rate from human to mosquito, *ϕ*_2_ is the progression rate from *I*_*T*_ to the latent stage, *b* is the number of vector bites per unit time, *ω*_1_ is the rate at which latent infected moves to Ebola undetected class, *ρ* is the rate at which treated Ebola-malaria individuals move to *E*_*M*_, *η*_*D*_ is the modification parameter of *I*_*D*_ in relation to *L*_*E*_. *η*_*T*_ is the modification parameter of *I*_*T*_, *η*_*J*_ is the modification parameter of *J*, *η*_1_ and *η*_2_ are the modification parameters of *E*_*EM*_ and *I*_*EM*_, respectively, *η*_*EM*_ is the modification parameter of *I*_*EM*_, and *θ* is the rate at which *J* individuals are discharged from the treatment centers.

### 3.1. Fractional Model

To capture the memory in the predictions of the Ebola-malaria coinfection model and also to check that both sides of the fractional equations have the exact dimensions, the coefficient 1/*α*^1−*σ*^ , comprised with the auxiliary parameter *α* [23, 24] is imposed on model (9). Hence, we suggest the following fractional-order model for the Ebola-malaria coinfection model under the ABC-fractional derivative:

(11) $$\begin{array}{c} \left\{\begin{array}{c} {\frac{1}{\alpha^{1-\sigma }}}^{ABC}D_{0_{+}}^{\sigma }S_{H}\left(\sigma \right)=\pi_{H}-\lambda_{E}S_{H}-\lambda_{M}S_{H}-\lambda_{EM}S_{H}-\mu S_{H}+\phi_{1}R_{M}+\alpha \theta J,\\ {\frac{1}{\alpha^{1-\sigma }}}^{ABC}D_{0_{+}}^{\sigma }L_{E}\left(\sigma \right)=\varepsilon_{1}\lambda_{E}S_{H}-\left(K_{E}+\sigma_{1}+\mu \right)L_{E}+\phi_{2}I_{T}+\left(1-\alpha \right)\theta J-\left(1-\rho \right)\phi_{3}I_{EM},\\ {\frac{1}{\alpha^{1-\sigma }}}^{ABC}D_{0_{+}}^{\sigma }I_{U}\left(\sigma \right)=\left(1-\varepsilon_{1}\right)\lambda_{E}S_{H}+\omega_{1}K_{E}L_{E}-\left(\gamma_{UE}+\mu +\delta_{UE}\right)I_{U},\\ {\frac{1}{\alpha^{1-\sigma }}}^{ABC}D_{0_{+}}^{\sigma }I_{D}\left(\sigma \right)=\left(1-\omega_{1}\right)K_{E}L_{E}-\left(\tau_{1}+\mu +\delta_{ED}+\sigma_{2}\right)I_{D}+\gamma_{UE}I_{U}+\tau_{4}E_{EM},\\ {\frac{1}{\alpha^{1-\sigma }}}^{ABC}D_{0_{+}}^{\sigma }I_{T}\left(\sigma \right)=\tau_{1}I_{D}-\left(\phi_{2}+\mu \right)I_{T},\\ {\frac{1}{\alpha^{1-\sigma }}}^{ABC}D_{0_{+}}^{\sigma }J\left(\sigma \right)=\sigma_{1}L_{E}+\sigma_{2}I_{D}-\left(\mu +\delta_{j}\right)J-\theta J,\\ {\frac{1}{\alpha^{1-\sigma }}}^{ABC}D_{0_{+}}^{\sigma }E_{M}\left(\sigma \right)=\varepsilon_{2}\lambda_{M}S_{H}-\left(K_{M}+\mu \right)E_{M}-\tau_{2}E_{M}+\rho \phi_{3}I_{EM},\\ {\frac{1}{\alpha^{1-\sigma }}}^{ABC}D_{0_{+}}^{\sigma }I_{M}\left(\sigma \right)=\left(1-\varepsilon_{2}\right)\lambda_{M}S_{H}+K_{M}E_{M}-\left(\tau_{3}+r+\delta_{IM}+\mu \right)I_{M},\\ {\frac{1}{\alpha^{1-\sigma }}}^{ABC}D_{0_{+}}^{\sigma }R_{M}\left(\sigma \right)=\tau_{2}E_{M}+\tau_{3}I_{M}+rI_{M}-\left(\phi_{1}+\mu \right)R_{M},\\ {\frac{1}{\alpha^{1-\sigma }}}^{ABC}D_{0_{+}}^{\sigma }E_{EM}\left(\sigma \right)=\varepsilon_{3}\lambda_{EM}S_{H}+\left(K_{EM}+\delta_{IEM}+\mu \right)E_{EM}-\tau_{4}E_{EM},\\ {\frac{1}{\alpha^{1-\sigma }}}^{ABC}D_{0_{+}}^{\sigma }I_{EM}\left(\sigma \right)=\left(1-\varepsilon_{3}\right)\lambda_{EM}S_{H}+K_{EM}E_{EM}-\left(\phi_{3}+\delta_{IEM}+\mu \right)I_{EM},\\ {\frac{1}{\alpha^{1-\sigma }}}^{ABC}D_{0_{+}}^{\sigma }S_{V}\left(\sigma \right)=\pi_{V}-\lambda_{V}S_{V}-\mu_{V}S_{V},\\ {\frac{1}{\alpha^{1-\sigma }}}^{ABC}D_{0_{+}}^{\sigma }E_{V}\left(\sigma \right)=\lambda_{V}S_{V}-\left(\sigma_{V}+\mu_{V}\right)E_{V},\\ {\frac{1}{\alpha^{1-\sigma }}}^{ABC}D_{0_{+}}^{\sigma }I_{V}\left(\sigma \right)=\sigma_{V}E_{V}-\mu_{V}I_{V}, \end{array}\right. \end{array}$$

where 0 < *σ* ≤ 1, with the following initial conditions: *S*_*H*_(0) = *S*_*H*_0__ ≥ 0, *L*_*E*_(0) = *L*_*E*_0__ ≥ 0, *I*_*U*_(0) = *I*_*U*_0__ ≥ 0, *I*_*D*_(0) = *I*_*D*_0__ ≥ 0, *I*_*T*_(0) = *I*_*T*_0__ ≥ 0, *J*(0) = *J*_0_ ≥ 0, *E*_*M*_(0) = *E*_*M*_0__ ≥ 0, *R*_*M*_(0) = *R*_*M*_0__ ≥ 0, *E*_*EM*_(0) = *E*_*EM*_0__ ≥ 0, *I*_*EM*_(0) = *I*_*EM*_0__ ≥ 0*S*_*V*_(0) = *S*_*V*_0__ ≥ 0, *E*_*V*_(0) = *E*_*V*_0__ ≥ 0, *I*_*V*_(0) = *I*_*V*_0__ ≥ 0, and *I*_*M*_(0) = *I*_*M*_0__ ≥ 0.

## 4. Existence and Uniqueness

It is important to determine whether or not such a dynamical problem exists before delving into any type of epidemiological simulations. Fortunately, the fixed point theory provides an ironclad guarantee for this evaluation's outcome. We attempt to apply the same idea in a perspective of the Banach and Krassnoselskii's fixed point theory to the stated model (11) to study existence and uniqueness results. In relation to the aforementioned requirement, we reformulate the considered model (11) as follows:

(12) D ABC0+σSHσ=ℵ1Δ∗∗,D ABC0+σLEσ=ℵ2Δ∗∗,D ABC0+σIUσ=ℵ3Δ∗∗,D ABC0+σIDσ=ℵ4Δ∗∗,D ABC0+σITσ=ℵ5Δ∗∗,D ABC0+σJσ=ℵ6Δ∗∗,D ABC0+σEMσ=ℵ7Δ∗∗,D ABC0+σIMσ=ℵ8Δ∗∗,D ABC0+σRMσ=ℵ9Δ∗∗,D ABC0+σEEMσ=ℵ10Δ∗∗,D ABC0+σIEMσ=ℵ11Δ∗∗,D ABC0+σSVσ=ℵ12Δ∗∗,D ABC0+σEVσ=ℵ13Δ∗∗,D ABC0+σIVσ=ℵ14Δ∗∗,

where Δ^∗∗^ = (*σ*, *S*_*H*_, *L*_*E*_, *I*_*U*_, *I*_*D*_, *I*_*T*_, *J*, *E*_*M*_, *I*_*M*_, *R*_*M*_, *E*_*EM*_, *I*_*EM*_, *S*_*V*_, *E*_*V*_, *I*_*V*_) and

(13) $$\begin{array}{c} \left\{\begin{array}{c} \begin{array}{c} {ℵ}_{1}\left(\Delta^{**}\right)=\pi_{H}-\lambda_{E}S_{H}-\lambda_{M}S_{H}-\lambda_{EM}S_{H}-\mu S_{H}+\phi_{1}R_{M}+\alpha \theta J,\\ {ℵ}_{2}\left(\Delta^{**}\right)=\varepsilon_{1}\lambda_{E}S_{H}{-}_{\left(K_{E}+\sigma_{1}+\mu \right)}L_{E}+\phi_{2}I_{T}+\left(1-\alpha \right)\theta J-\left(1-\rho \right)\phi_{3}I_{EM},\\ {ℵ}_{3}\left(\Delta^{**}\right)=\left(1-\varepsilon_{1}\right)\lambda_{E}S_{H}{+}_{\omega_{1}K_{E}}L_{E}-\left(\gamma_{UE}+\mu +\delta_{UE}\right)I_{U},\\ {ℵ}_{4}\left(\Delta^{**}\right)=\left(1-\omega_{1}\right)K_{E}L_{E}-\left(\tau_{1}+\mu +\delta_{ED}+\sigma_{2}\right)I_{D}+\gamma_{UE}I_{U}+\tau_{4}E_{EM},\\ {ℵ}_{5}\left(\Delta^{**}\right)=\tau_{1}I_{D}-\left(\phi_{2}+\mu \right)I_{T},\\ {ℵ}_{6}\left(\Delta^{**}\right)=\sigma_{1}L_{E}{+}_{\sigma_{2}}I_{D}-\left(\mu +\delta_{j}\right)J-\theta J,\\ {ℵ}_{7}\left(\Delta^{**}\right)=\varepsilon_{2}\lambda_{M}S_{H}-\left(K_{M}+\mu \right)E_{M}-\tau_{2}E_{M}+\rho \phi_{3}I_{EM},\\ {ℵ}_{8}\left(\Delta^{**}\right)=\left(1-\varepsilon_{2}\right)\lambda_{M}S_{H}{+}_{K_{M}}E_{M}-\left(\tau_{3}+r+\delta_{IM}+\mu \right)I_{M},\\ {ℵ}_{9}\left(\Delta^{**}\right)=\tau_{2}E_{M}+\tau_{3}I_{M}+rI_{M}-\left(\phi_{1}+\mu \right)R_{M},\\ {ℵ}_{10}\left(\Delta^{**}\right)=\varepsilon_{3}\lambda_{EM}S_{H}+\left(K_{EM}+\delta_{IEM}+\mu \right)E_{EM}-\tau_{4}E_{EM},\\ {ℵ}_{11}\left(\Delta^{**}\right)=\left(1-\varepsilon_{3}\right)\lambda_{EM}S_{H}{+}_{K_{EM}}E_{EM}-\left(\phi_{3}+\delta_{IEM}+\mu \right)I_{EM},\\ {ℵ}_{12}\left(\Delta^{**}\right)=\pi_{V}-\lambda_{V}S_{V}-\mu_{V}S_{V},\\ {ℵ}_{13}\left(\Delta^{**}\right)=\lambda_{V}S_{V}-\left(\sigma_{V}+\mu_{V}\right)E_{V},\\ {ℵ}_{14}\left(\Delta^{**}\right)=\sigma_{V}E_{V}-\mu_{V}I_{V}. \end{array} \end{array}\right. \end{array}$$

For simplicity we write the model (11) in the form;

(14) D ABCσωWσ=Ψσ,Wσ,σ∈0,η,W0=W0,

where

(15) $$\begin{array}{c} \left\{\begin{array}{c} \begin{array}{c} W={\left(S_{H},L_{E},I_{U},I_{D},I_{T},J,E_{M},I_{M},R_{M},E_{EM},I_{EM},S_{V},E_{V},I_{V}\right)}^{T},\\ W\left(0\right)={\left(T_{1},T_{2}\right)}^{T},\\ \Psi \left(\sigma ,W\left(\sigma \right)\right)={ℵ}_{i}{\left(\Delta^{**}\right)}^{T},\\ i=1,2,3,\cdots ,14, \end{array} \end{array}\right. \end{array}$$

where (.)^*T*^ presents the transpose of the vectors, *T*_1_ = (*S*_*H*_(0), *L*_*E*_(0), *I*_*U*_(0), *I*_*D*_(0), *I*_*T*_(0), *J*(0), *E*_*M*_(0)), and *T*_2_ = (*I*_*M*_(0), *R*_*M*_(0), *E*_*EM*_(0), *I*_*EM*_(0), *S*_*V*_(0), *E*_*V*_(0), *I*_*V*_(0))^*T*^. From Lemma 2.2, the system (14) is equal to the following fractional integral equation;

(16) $$\begin{array}{c} \begin{array}{c} \begin{array}{c} W\left(\sigma \right)=W_{0}+\frac{1-\omega }{\nabla \left(\omega \right)}\Psi \left(\sigma ,W\left(\sigma \right)\right)+\frac{\omega }{\nabla \left(\omega \right)\Gamma \left(\omega \right)}\int_{0}^{\sigma }\Psi \left(s,W\left(s\right)\right){\left(\sigma -s\right)}^{\omega -1}ds. \end{array} \end{array} \end{array}$$

Let us say *B* = *C*([0, *η*]) is the Banach space, supposing that the following assumptions hold;

(F_1_) There exist a nonnegative constant Y, Z, and *a* ∈ [0, 1) such that

(17) $$\begin{array}{c} \Psi \left(\sigma ,W\left(\sigma \right)\right)\leq Y{\left|W\right|}^{a}+Z. \end{array}$$

(F_2_) There exist a nonnegative constant **L**_*μ*_ > 0 for all **W**, **W**^∗^ ∈ **B** then

(18) $$\begin{array}{c} \left|\Psi \left(\sigma ,W\left(\sigma \right)\right)-\Psi \left(\sigma ,W^{*}\left(\sigma \right)\right)\right|\leq L_{\mu }\left[\left|W-W^{*}\right|\right]. \end{array}$$

Also, let us define operator **A**_*p*_ : **B**⟶**B** such that

(19) $$\begin{array}{c} A_{p}W\left(\sigma \right)=\Omega_{1}W\left(\sigma \right)+\Omega_{2}W\left(\sigma \right), \end{array}$$

basically, we let

(20) $$\begin{array}{c} \left\{\begin{array}{c} \begin{array}{c} \Omega_{1}W\left(\sigma \right)=W_{0}+\frac{1-\omega }{\nabla \left(\omega \right)}\Psi \left(\sigma ,W\left(\sigma \right)\right),\\ \Omega_{2}W\left(\sigma \right)=\frac{\omega }{\nabla \left(\omega \right)\Gamma \left(\omega \right)}\int_{0}^{\sigma }\Psi \left(s,W\left(s\right)\right){\left(\sigma -s\right)}^{\omega -1}ds. \end{array} \end{array}\right. \end{array}$$

From this knowledge, equation (16) can be written as;

(21) $$\begin{array}{c} \begin{array}{c} \begin{array}{c} A_{p}W\left(\sigma \right)=W_{0}+\frac{\left(1-\omega \right)}{\nabla \left(\omega \right)}\Psi \left(\sigma ,W\left(\sigma \right)\right)+\frac{\omega }{\nabla \left(\omega \right)\Gamma \left(\omega \right)}\int_{0}^{\sigma }\Psi \left(s,W\left(s\right)\right){\left(\sigma -s\right)}^{\omega -1}ds. \end{array} \end{array} \end{array}$$

**Theorem 1 .**

Suppose that (F_1_) and (F_2_) hold, such that, ((1 − *ω*)/∇(*ω*))**L**_*μ*_ < 1, then the Ebola-malaria co-infection model (14) has at least one solution.

**Proof**

We divide the proof into two steps:

Step 1. We prove that operator *Ω*_1_ is contraction. Then, let **W**^∗^ ∈ *Π*, where *Π* = {**W** ∈ *B* : ‖**W**‖ ≤ *ρ*, *ρ* > 0} is a close convex set, thus

(22) $$\begin{array}{c} \left|\Omega_{1}\left(W\right)-\Omega_{1}\left(W^{*}\right)\right|=\frac{\left(1-\omega \right)}{\nabla \left(\omega \right)}\underset{\omega \in \left[0,\eta \right]}{\max}\left|\Psi \left(\sigma ,W\left(\sigma \right)\right)-\Psi \left(\sigma ,W^{*}\left(\sigma \right)\right)\right|,\leq \frac{\left(1-\omega \right)}{\nabla \left(\omega \right)}L_{\mu }\left\|W-W^{*}\right\|. \end{array}$$

Hence *Ω*_1_ is contraction.

Step 2. We prove that *Ω*_2_ is compact and also continuous, for all **W** ∈ *Π*, then *Ω*_2_ will be continuous as **W** is continuous; thus,

(23) $$\begin{array}{c} \left\|\Omega_{2}\left(W\right)\right\|=\underset{\omega \in \left[0,\eta \right]}{\max}\left|\frac{\omega }{\nabla \left(\omega \right)\Gamma \left(\omega \right)}\int_{0}^{\sigma }\Psi \left(s,W\left(s\right)\right){\left(\sigma -s\right)}^{\omega -1}\right|ds,\leq \frac{\omega }{\nabla \left(\omega \right)\Gamma \left(\omega \right)}\int_{0}^{\eta }\left|{\left(\eta -s\right)}^{\omega -1}\right|\left|\Psi \left(s,W\left(s\right)\right)\right|ds.\leq \frac{\eta^{\omega }}{\nabla \left(\omega \right)\Gamma \left(\omega \right)}\left[Y{\left|W\right|}^{a}+Z\right]. \end{array}$$

Hence *Ω*_2_ is boundedness. For equicontinuous, let *σ*_1_ and *σ*_2_ ∈ [0, *η*], such that

(24) $$\begin{array}{c} \left|\left(\Omega_{2}W\right)\left(\sigma_{1}\right)-\left(\Omega_{2}W\right)\left(\sigma_{2}\right)\right|=\left|\frac{\omega }{\nabla \left(\omega \right)\Gamma \left(\omega \right)}\right|\int_{0}^{\sigma_{1}}\Psi \left(s,W\left(s\right)\right){\left(\sigma_{1}-s\right)}^{\omega -1}ds-\int_{0}^{\sigma_{2}}\Psi \left(s,W\left(s\right)\right)\left.{\left(\sigma_{2}-s\right)}^{\omega -1}\right|ds\leq \frac{\left[Y{\left|W\right|}^{a}+Z\right]}{\nabla \left(\omega \right)\Gamma \left(\omega \right)}\left[\sigma_{1}^{\omega }-\sigma_{2}^{\omega }\right]. \end{array}$$

As *σ*_1_⟶*σ*_2_, then |(*Ω*_2_**W**)(*σ*_1_) − (*Ω*_2_**W**)(*σ*_2_)|⟶0 which make operator *Ω*_2_ an equicontinuous and compact by the Arzela-Ascoli theorem. Therefore the existence for the Ebola-malaria co-infection model (11) is proved.

**Theorem 2 .**

Suppose that ∃ a nonnegative integer *Λ* > 0 such that

(25) $$\begin{array}{c} \begin{array}{c} \begin{array}{c} \Lambda =\left[\frac{\left(1-\omega \right)}{\nabla \left(\omega \right)}L_{\mu }+\frac{\eta^{\omega }}{\nabla \left(\omega \right)\Gamma \left(\omega \right)}L_{\mu }\right]<1, \end{array} \end{array} \end{array}$$

then operator **A**_*p*_ has a unique fixed point.

**Proof**

Let **W**, **W**^∗^ ∈ **B**, then we say

(26) $$\begin{array}{c} \left\|A_{p}W-A_{p}W^{*}\right\|\leq \left\|\Omega_{1}W-\Omega_{1}W^{*}\right\|+\left\|\Omega_{2}W-\Omega_{2}W^{*}\right\|,\leq \left.\frac{\left(1-\omega \right)}{\nabla \left(\omega \right)}\right|\underset{\omega \in \left[0,\eta \right]}{\max}\left|\Psi \left(\sigma ,W\left(\sigma \right)\right)-\Psi \left(\sigma ,W^{*}\left(\sigma \right)\right)\right|+\frac{\omega }{\nabla \left(\omega \right)\Gamma \left(\omega \right)}\underset{\omega \in \left[0,\eta \right]}{\max}\left|\int_{0}^{\sigma }\Psi \left(s,W\left(s\right)\right){\left(\sigma -s\right)}^{\omega -1}ds-\int_{0}^{\sigma }\Psi \left(s,W^{*}\left(s\right)\right){\left(\sigma -s\right)}^{\omega -1}\right|ds,\leq \left[\frac{\left(1-\omega \right)}{\nabla \left(\omega \right)}L_{\mu }+\frac{\eta^{\omega }}{\nabla \left(\omega \right)\Gamma \left(\omega \right)}L_{\mu }\right]\left\|W-W^{*}\right\|,=\Lambda \left\|W-W^{*}\right\|. \end{array}$$

Hence, by the Banach contraction principle, **A**_*p*_ has a unique fixed point. Consequently, the Ebola-malaria co-infection model (11) has unique solution.

## 5. Hyers-Ulam Stability

In the context of differential equations, stability is crucial. The Hyers-Ulam (HU) type of stability has emerged as one of the most intriguing types of stability in recent years. Here, we use HU type stability to examine a theoretical model of Ebola and malaria transmission.

**Definition 3 .**

The Ebola-malaria coinfection model (11) is HU stable if for *δ* > 0 and letting *W* ∈ *B* be any solution of below inequality

(27) D ABCσωWσ−Ψσ,Wσ≤δ,∀σ∈0,η;

and with a unique solution **W**^∗^ of problem (14) with a positive constant *λ*_*q*_ > 0, such that,

(28) $$\begin{array}{c} \begin{array}{c} \begin{array}{c} \left\|W-W^{*}\right\|\leq \lambda_{q}\delta ,\forall \sigma \in \left[0,\eta \right]. \end{array} \end{array} \end{array}$$

**Definition 4 .**

Given a function *ϕ* ∈ *C*([0, *η*], *R*), such that *ϕ*(0) = 0 for any solution **W** of (27) and **W**^∗^ be a unique solution of (14), then

(29) $$\begin{array}{c} \left\|W-W^{*}\right\|\leq \phi \left(\delta \right), \end{array}$$

then the Ebola-malaria co-infection model (14) is generalized HU stable.

**Remark 1 .**

Suppose *χ*(*σ*) ∈ *C*([0, *η*], *R*), we say **W** ∈ **B** satisfies inequality (27) suppose that,

- |*χ*(*σ*)| ≤ *δ*, for all *σ* ∈ [0, *η*]
- _ _^*ABC*^*D*_*σ*_^*ω*^*W*(*σ*) = Ψ(*σ*, *W*(*σ*)) + *χ*(*σ*), ∀*σ* ∈ [0, *η*].

Now, we consider the resulting perturbation equation of system (14) as follows;

(30) D ABCσωWσ=Ψσ,Wσ+χσ,W0=W0.

The below Lemma is needed to help us get our results.

**Lemma 4 .**

From equation (30), we say the following result hold. Thus,

(31) $$\begin{array}{c} \left|W\left(\sigma \right)-A_{p}\Psi \left(\sigma ,W\left(\sigma \right)\right)\right|\leq \left[\frac{\left(1-\omega \right)}{\nabla \left(\omega \right)}+\frac{\eta^{\omega }}{\nabla \left(\omega \right)\Gamma \left(\omega \right)}\right]\delta . \end{array}$$

**Proof**

Consider Lemma 2.2 relatively, solution for equation (14) is given as;

(32) Wσ=W0+I ABCσωΨσ,Wσ+I ABCσωχσ.

Now, with the help of equation (21), we deduce that

(33) $$\begin{array}{c} \left|W\left(\sigma \right)-A_{p}\Psi \left(\sigma ,W\left(\sigma \right)\right)\right|\leq \left[\frac{\left(1-\omega \right)}{\nabla \left(\omega \right)}\left|\chi \left(\sigma \right)\right|+\frac{\eta^{\omega }}{\nabla \left(\omega \right)\Gamma \left(\omega \right)}\int_{0}^{\sigma }{\left(\sigma -s\right)}^{1-\omega }\left|\chi \left(\sigma \right)\right|ds\right]\leq \left[\frac{\left(1-\omega \right)}{\nabla \left(\omega \right)}+\frac{\eta^{\omega }}{\nabla \left(\omega \right)\Gamma \left(\omega \right)}\right]\delta . \end{array}$$

**Theorem 3 .**

Suppose that the Ebola-malaria co-infection model (14) is Ulam-Hyers stable, if there exist *Λ* = [((1 − *ω*)/∇(*ω*))**L**_*μ*_ + (*η*^*ω*^/∇(*ω*)Γ(*ω*))**L**_*μ*_] < 1.

**Proof**

With the help from the Lemma 5.1, let **W** ∈ **B** be any solution and **W**^∗^ ∈ **B** be a unique solution for considered problem (14), then

(34) $$\begin{array}{c} \left|W\left(\sigma \right)-W^{*}\left(\sigma \right)\right|=\left|W\left(\sigma \right)-A_{p}W^{*}\left(\sigma \right)\right|\leq \left|W\left(\sigma \right)-A_{p}W\left(\sigma \right)\right|+\left|A_{p}W\left(\sigma \right)-A_{p}W^{*}\left(\sigma \right)\right|\leq \left[\frac{\left(1-\omega \right)}{\nabla \left(\omega \right)}+\frac{\eta^{\omega }}{\nabla \left(\omega \right)\Gamma \left(\omega \right)}\right]\delta +\left[\frac{\left(1-\omega \right)}{\nabla \left(\omega \right)}L_{\mu }+\frac{\eta^{\omega }}{\nabla \left(\omega \right)\Gamma \left(\omega \right)}L_{\mu }\right]\left\|W-W^{*}\right\|. \end{array}$$

Thus,

(35) $$\begin{array}{c} \left\|W\left(\sigma \right)-W^{*}\left(\sigma \right)\right\|\leq \frac{\left[\left(\left(1-\omega \right)/\nabla \left(\omega \right)\right)+\left(\eta^{\omega }/\nabla \left(\omega \right)\Gamma \left(\omega \right)\right)\right]}{1-\left[\left(\left(1-\omega \right)/\nabla \left(\omega \right)\right)L_{\mu }+\left(\eta^{\omega }/\nabla \left(\omega \right)\Gamma \left(\omega \right)\right)L_{\mu }\right]}\delta . \end{array}$$

Hence, we conclude that, the Ebola-malaria co-infection model (14) is HU stable. Consequently, the Ebola-malaria co-infection model (14) is HU generalized stable.

**Definition 5 .**

The problem (14) is Hyers-Ulam-Rassias (HUR) stable given that the function *ξ*(*σ*) ∈ *C*([0, 1], *R*), *δ* > 0 and letting **W** ∈ **B** be any solution of the below inequality

(36) D ABCωσWσ−Ψσ,Wσ≤ξσδ,∀σ∈0,η;

and also ∃ unique solution **W**^∗^ of problem (14) with a positive constant *λ*_*q*_ > 0 then,

(37) $$\begin{array}{c} \left\|W-W^{*}\right\|\leq \lambda_{q}\xi \left(\sigma \right)\delta ,\forall \sigma \in \left[0,\eta \right]. \end{array}$$

**Definition 6 .**

Given a function *ν* ∈ *C*([0, *η*], *R*), with *λ*_*q*,*ν*_ and *δ* > 0, for all **W** of equation (36) and **W**^∗^ be a unique solution of (14), then

(38) $$\begin{array}{c} \begin{array}{c} \begin{array}{c} \left\|W-W^{*}\right\|\leq \lambda_{q,\nu }\nu \left(\sigma \right),\forall \sigma \in \left[0,\eta \right], \end{array} \end{array} \end{array}$$

then system (14) is HUR generalized stable.

**Remark 2 .**

Suppose *μ*(*σ*) ∈ *C*([0, 1], *R*), we say *W* ∈ *B* satisfies inequality (36), suppose that,

- |*μ*(*σ*)| ≤ *δν*(*σ*), ∀*σ* ∈ [0, *η*].
- _*ω*_^*ABC*^*D*_*ω*_^*σ*^**W**(*σ*) = Ψ(*σ*, **W**(*σ*)) + *μ*(*σ*), ∀*σ* ∈ [0, *η*].

Now, we consider the resulting perturbation equation of system (14) as follows:

(39) D ABCσωWσ=Ψσ,Wσ+μσ,W0=W0.

**Lemma 5 .**

From equation (39), we say the following result hold. Thus,

(40) $$\begin{array}{c} \left|W\left(\sigma \right)-A_{p}\Psi \left(\sigma ,W\left(\sigma \right)\right)\right|\leq \left[\frac{\left(1-\omega \right)}{\nabla \left(\omega \right)}+\frac{\eta^{\omega }}{\nabla \left(\omega \right)\Gamma \left(\omega \right)}\right]\mu \left(\sigma \right)\delta . \end{array}$$

**Proof**

Consider Lemma 2.2 relatively, solution for equation (39) is given as;

(41) Wσ=W0+I ABCσωΨσ,Wσ+I ABCσωμσ.

Now, with the help of (21), we deduce that

(42) $$\begin{array}{c} \left|W\left(\sigma \right)-A_{p}\Psi \left(\sigma ,W\left(\sigma \right)\right)\right|\leq \left[\frac{\left(1-\omega \right)}{\nabla \left(\omega \right)}\left|\nu \left(\sigma \right)\right|+\frac{\eta^{\omega }}{\nabla \left(\omega \right)\Gamma \left(\omega \right)}\int_{0}^{\sigma }{\left(\sigma -s\right)}^{1-\omega }\left|\mu \left(\sigma \right)\right|ds\right]\leq \left[\frac{\left(1-\omega \right)}{\nabla \left(\omega \right)}+\frac{\eta^{\omega }}{\nabla \left(\omega \right)\Gamma \left(\omega \right)}\right]\mu \left(\sigma \right)\delta . \end{array}$$

**Theorem 4 .**

Suppose that the Ebola-malaria co-infection (11) is HUR stable if ∃

(43) $$\begin{array}{c} \Lambda =\left[\frac{\left(1-\omega \right)}{\nabla \left(\omega \right)}L_{\mu }+\frac{\eta^{\omega }}{\nabla \left(\omega \right)\Gamma \left(\omega \right)}L_{\mu }\right]<1. \end{array}$$

**Proof**

With the help from the Lemma 5.3, let *W* ∈ *B* be any solution and *W*^∗^ ∈ *B* be a unique solution for considered problem (14), then

(44) $$\begin{array}{c} \left|W\left(\sigma \right)-W^{*}\left(\sigma \right)\right|=\left|W\left(\sigma \right)-A_{p}W^{*}\left(\sigma \right)\right|\leq \left|W\left(\sigma \right)-A_{p}W\left(\sigma \right)\right|+\left|A_{p}W\left(\sigma \right)-A_{p}W^{*}\left(\sigma \right)\right|\leq \left[\frac{\left(1-\omega \right)}{\nabla \left(\omega \right)}+\frac{\eta^{\omega }}{\nabla \left(\omega \right)\Gamma \left(\omega \right)}\right]\nu \left(\sigma \right)\delta +\left[\frac{\left(1-\omega \right)}{\nabla \left(\omega \right)}L_{\mu }+\frac{\eta^{\omega }}{\nabla \left(\omega \right)\Gamma \left(\omega \right)}L_{\mu }\right]\left\|W-W^{*}\right\|. \end{array}$$

Thus,

(45) $$\begin{array}{c} \left\|W\left(\sigma \right)-W^{*}\left(\sigma \right)\right\|\leq \frac{\left[\left(\left(1-\omega \right)/\nabla \left(\omega \right)\right)+\left(\eta^{\omega }/\nabla \left(\omega \right)\Gamma \left(\omega \right)\right)\right]}{1-\left[\left(\left(1-\omega \right)/\nabla \left(\omega \right)\right)L_{\mu }+\left(\eta^{\omega }/\nabla \left(\omega \right)\Gamma \left(\omega \right)\right)L_{\mu }\right]}\nu \left(\sigma \right)\delta . \end{array}$$

Hence, we conclude that, the Ebola-malaria coinfection (11) is HUR stable. Consequently, the Ebola-malaria coinfection model (11) is generalized HUR stable.

## 6. Numerical Scheme

Here we provide the numerical schemes for the two-step Lagrange interpolation used in our considered ABC-fractional operator model of the Ebola-malaria coinfection. By using the initial condition and the operator _ _^*ABC*^*I*_0_^*ω*^, we transform the Ebola-malaria co-infection (14) into a system of fractional integral equations, as shown below.

(46) SHσ−SH0=I ABC0ωℵ1σ,SHσ,LEσ−LE0=I ABC0ωℵ2σ,LEσ,IUσ−IU0=I ABC0ωℵ3σ,IUσ,IDσ−ID0=I ABC0ωℵ4σ,IDσ,ITσ−IT0=I ABC0ωℵ5σ,ITσ,Jσ−J0=I ABC0ωℵ6σ,Jσ,EMσ−EM0=I ABC0ωℵ7σ,EMσ,IMσ−IM0=I ABC0ωℵ8σ,IMσ,RMσ−RM0=I ABC0ωℵ9σ,RMσ,EEMσ−EEM0=I ABC0ωℵ10σ,EEMσ,IEMσ−IEM0=I ABC0ωℵ11σ,IEMσ,SVσ−SV0=I ABC0ωℵ12σ,SVσ,EVσ−EV0=I ABC0ωℵ13σ,EVσ,IVσ−IV0=I ABC0ωℵ14σ,IVσ,

which we can easily get the following:

(47) $$\begin{array}{c} S_{H}\left(\sigma \right)=S_{H}\left(0\right)+\frac{1-\omega }{\nabla \left(\omega \right)}{ℵ}_{1}\left(\sigma ,S_{H}\left(\sigma \right)\right)+\frac{\omega }{\nabla \left(\omega \right)\Gamma \left(\omega \right)}\int_{0}^{\sigma }{ℵ}_{1}\left(s,S_{H}\left(s\right)\right){\left(\sigma -s\right)}^{\omega -1}ds,\\ L_{E}\left(\sigma \right)=L_{E}\left(0\right)+\frac{1-\omega }{\nabla \left(\omega \right)}{ℵ}_{2}\left(\sigma ,L_{E}\left(\sigma \right)\right)+\frac{\omega }{\nabla \left(\omega \right)\Gamma \left(\omega \right)}\int_{0}^{\sigma }{ℵ}_{2}\left(s,L_{E}\left(s\right)\right){\left(\sigma -s\right)}^{\omega -1}ds,\\ I_{U}\left(\sigma \right)=I_{U}\left(0\right)+\frac{1-\omega }{\nabla \left(\omega \right)}{ℵ}_{3}\left(\sigma ,I_{U}\left(\sigma \right)\right)+\frac{\omega }{\nabla \left(\omega \right)\Gamma \left(\omega \right)}\int_{0}^{\sigma }{ℵ}_{3}\left(s,I_{U}\left(s\right)\right){\left(\sigma -s\right)}^{\omega -1}ds,\\ I_{D}\left(\sigma \right)=I_{D}\left(0\right)+\frac{1-\omega }{\nabla \left(\omega \right)}{ℵ}_{4}\left(\sigma ,I_{D}\left(\sigma \right)\right)+\frac{\omega }{\nabla \left(\omega \right)\Gamma \left(\omega \right)}\int_{0}^{\sigma }{ℵ}_{4}\left(s,I_{D}\left(s\right)\right){\left(\sigma -s\right)}^{\omega -1}ds,\\ I_{T}\left(\sigma \right)=I_{T}\left(0\right)+\frac{1-\omega }{\nabla \left(\omega \right)}{ℵ}_{5}\left(\sigma ,I_{T}\left(\sigma \right)\right)+\frac{\omega }{\nabla \left(\omega \right)\Gamma \left(\omega \right)}\int_{0}^{\sigma }{ℵ}_{5}\left(s,I_{T}\left(s\right)\right){\left(\sigma -s\right)}^{\omega -1}ds,\\ J\left(\sigma \right)=J\left(0\right)+\frac{1-\omega }{\nabla \left(\omega \right)}{ℵ}_{6}\left(\sigma ,J\left(\sigma \right)\right)+\frac{\omega }{\nabla \left(\omega \right)\Gamma \left(\omega \right)}\int_{0}^{\sigma }{ℵ}_{6}\left(s,J\left(s\right)\right){\left(\sigma -s\right)}^{\omega -1}ds,\\ E_{M}\left(\sigma \right)=E_{M}\left(0\right)+\frac{1-\omega }{\nabla \left(\omega \right)}{ℵ}_{7}\left(\sigma ,E_{M}\left(\sigma \right)\right)+\frac{\omega }{\nabla \left(\omega \right)\Gamma \left(\omega \right)}\int_{0}^{\sigma }{ℵ}_{7}\left(s,E_{M}\left(s\right)\right){\left(\sigma -s\right)}^{\omega -1}ds,\\ I_{M}\left(\sigma \right)=I_{M}\left(0\right)+\frac{1-\omega }{\nabla \left(\omega \right)}{ℵ}_{8}\left(\sigma ,I_{M}\left(\sigma \right)\right)+\frac{\omega }{\nabla \left(\omega \right)\Gamma \left(\omega \right)}\int_{0}^{\sigma }{ℵ}_{8}\left(s,I_{M}\left(s\right)\right){\left(\sigma -s\right)}^{\omega -1}ds,\\ R_{M}\left(\sigma \right)=R_{M}\left(0\right)+\frac{1-\omega }{\nabla \left(\omega \right)}{ℵ}_{9}\left(\sigma ,R_{M}\left(\sigma \right)\right)+\frac{\omega }{\nabla \left(\omega \right)\Gamma \left(\omega \right)}\int_{0}^{\sigma }{ℵ}_{9}\left(s,R_{M}\left(s\right)\right){\left(\sigma -s\right)}^{\omega -1}ds,\\ E_{EM}\left(\sigma \right)=E_{EM}\left(0\right)+\frac{1-\omega }{\nabla \left(\omega \right)}{ℵ}_{10}\left(\sigma ,E_{EM}\left(\sigma \right)\right)+\frac{\omega }{\nabla \left(\omega \right)\Gamma \left(\omega \right)}\int_{0}^{\sigma }{ℵ}_{11}\left(s,E_{EM}\left(s\right)\right){\left(\sigma -s\right)}^{\omega -1}ds,\\ I_{EM}\left(\sigma \right)=I_{EM}\left(0\right)+\frac{1-\omega }{\nabla \left(\omega \right)}{ℵ}_{11}\left(\sigma ,I_{EM}\left(\sigma \right)\right)+\frac{\omega }{\nabla \left(\omega \right)\Gamma \left(\omega \right)}\int_{0}^{\sigma }{ℵ}_{11}\left(s,I_{EM}\left(s\right)\right){\left(\sigma -s\right)}^{\omega -1}ds,\\ S_{V}\left(\sigma \right)=S_{V}\left(0\right)+\frac{1-\omega }{\nabla \left(\omega \right)}{ℵ}_{12}\left(\sigma ,S_{V}\left(\sigma \right)\right)+\frac{\omega }{\nabla \left(\omega \right)\Gamma \left(\omega \right)}\int_{0}^{\sigma }{ℵ}_{12}\left(s,S_{V}\left(s\right)\right){\left(\sigma -s\right)}^{\omega -1}ds,\\ E_{V}\left(\sigma \right)=E_{V}\left(0\right)+\frac{1-\omega }{\nabla \left(\omega \right)}{ℵ}_{13}\left(\sigma ,E_{V}\left(\sigma \right)\right)+\frac{\omega }{\nabla \left(\omega \right)\Gamma \left(\omega \right)}\int_{0}^{\sigma }{ℵ}_{13}\left(s,E_{V}\left(s\right)\right){\left(\sigma -s\right)}^{\omega -1}ds,\\ I_{V}\left(\sigma \right)=I_{V}\left(0\right)+\frac{1-\omega }{\nabla \left(\omega \right)}{ℵ}_{14}\left(\sigma ,I_{V}\left(\sigma \right)\right)+\frac{\omega }{\nabla \left(\omega \right)\Gamma \left(\omega \right)}\int_{0}^{\sigma }{ℵ}_{14}\left(s,I_{V}\left(s\right)\right){\left(\sigma -s\right)}^{\omega -1}ds. \end{array}$$

Consider the ABC derivative under the Cauchy problem, and the ABC integral of Lemma 2.2 can be replicated using the fundamental theory of calculus.

(48) $$\begin{array}{c} \begin{array}{c} \Theta \left(\sigma \right)=\Theta_{0}+\frac{1-\omega }{\nabla \left(\omega \right)}ℵ\left(\sigma ,\Theta \left(\sigma \right)\right)+\frac{\omega }{\nabla \left(\omega \right)\Gamma \left(\omega \right)}\int_{0}^{\sigma }ℵ\left(\sigma ,\Theta \left(\sigma \right)\right){\left(\sigma -s\right)}^{\omega -1}ds. \end{array} \end{array}$$

Taking the point *σ*_(*z*^∗^ + 1)_ = (*z*^∗^ + 1)*h* and *σ*_*z*^∗^_ = *z*^∗^*h*, *z*^∗^ = 0, 1, 2, ⋯, with *h* being the time step, we can simply deduce

(49) $$\begin{array}{c} \Theta \left(\sigma_{z^{*}+1}\right)=\Theta_{0}+\frac{1-\omega }{\nabla \left(\omega \right)}ℵ\left(\sigma ,\Theta \left(\sigma \right)\right)+\frac{\omega }{\nabla \left(\omega \right)\Gamma \left(\omega \right)}\int_{0}^{\sigma }ℵ\left(s,\Theta \left(s\right)\right){\left(\sigma -s\right)}^{\omega -1}ds,=\Theta_{0}+\frac{1-\omega }{\nabla \left(\omega \right)}ℵ\left(\sigma_{z^{*}},\Theta \left(\sigma_{z^{*}}\right)\right)+\frac{\omega }{\nabla \left(\omega \right)\Gamma \left(\omega \right)}\int_{0}^{\sigma_{z^{*}+1}}ℵ\left(\theta ,\Theta \left(\theta \right)\right){\left(\sigma_{z^{*}+1}-\theta \right)}^{\omega -1}d\theta ,=\Theta_{0}+\frac{1-\omega }{\nabla \left(\omega \right)}ℵ\left(\sigma_{z^{*}},\Theta \left(\sigma_{z^{*}}\right)\right)+\frac{\omega }{\nabla \left(\omega \right)\Gamma \left(\omega \right)}\overset{z^{*}}{\underset{r_{*}=0}{\sum }}\int_{\sigma_{r_{*}}}^{\sigma_{r_{*}+1}}ℵ\left(\theta ,\Theta \left(\theta \right)\right){\left(\sigma_{z^{*}+1}-\theta \right)}^{\omega -1}d\theta . \end{array}$$

Having the interval of [*σ*_*z*^∗^_, *σ*_(*z*^∗^ + 1)_], the two term Lagrange polynomial is given as follows:

(50) $$\begin{array}{c} \gamma_{r_{*}}\left(\theta \right)=\frac{\theta -\sigma_{r_{*}-1}}{\sigma_{r_{*}}-\sigma_{r_{*}-1}}ℵ\left(\sigma_{r_{*}},\Theta \left(\sigma_{r_{*}}\right)\right)-\frac{\theta -\sigma_{r_{*}}}{\sigma_{r_{*}}-\sigma_{r_{*}-1}}ℵ\left(\sigma_{r_{*}-1},\Theta \left(\sigma_{r_{*}-1}\right)\right),=\frac{ℵ\left(\sigma_{r_{*}},\Theta \left(\sigma_{r_{*}}\right)\right)}{h}\left(\theta -\sigma_{r_{*}-1}\right)-\frac{ℵ\left(\sigma_{r_{*}-1},\Theta \left(\sigma_{r_{*}-1}\right)\right)}{h}\left(\theta -\sigma_{r_{*}}\right),≃\frac{ℵ\left(\sigma_{r_{*}},\Theta_{r_{*}}\right)}{h}\left(\theta -\sigma_{r_{*}-1}\right)-\frac{ℵ\left(\sigma_{r_{*}-1},\Theta_{r_{*}-1}\right)}{h}\left(\theta -\sigma_{r_{*}}\right). \end{array}$$

Taking the approximation solution of (50) into (49);

(51) $$\begin{array}{c} \Theta \left(\sigma_{z^{*}+1}\right)=\Theta_{0}+\frac{1-\omega }{\nabla \left(\omega \right)}ℵ\left(\sigma_{z^{*}},\Theta \left(\sigma_{z^{*}}\right)\right)+\frac{\omega }{\nabla \left(\omega \right)\Gamma \left(\omega \right)}\times \overset{z^{*}}{\underset{r_{*}=0}{\sum }}\left[\frac{ℵ\left(\sigma_{r_{*}},\Theta_{r_{*}}\right)}{h}\int_{\sigma_{r_{*}}}^{\sigma_{r_{*}+1}}\left(\theta -\sigma_{r_{*}-1}\right){\left(\sigma_{z^{*}+1}-\sigma \right)}^{\omega -1}d\theta -\frac{ℵ\left(\sigma_{r_{*}-1},\Theta_{r_{*}-1}\right)}{h}\int_{\sigma_{r_{*}}}^{\sigma_{r_{*}+1}}\left(\theta -\sigma_{r_{*}}\right){\left(\sigma_{z^{*}+1}-\sigma \right)}^{\omega -1}d\theta \right]. \end{array}$$

Solving the integral equations in the (51), let us take:

(52) $$\begin{array}{c} \begin{array}{c} Y_{\omega ,r_{*},1}=\int_{\sigma_{r_{*}}}^{\sigma_{r_{*}+1}}\left(\theta -\sigma_{r_{*}-1}\right){\left(\sigma_{z^{*}+1}-\sigma \right)}^{\omega -1}d\theta ,\\ Y_{\omega ,r_{*},2}=\int_{\sigma_{r_{*}}}^{\sigma_{r_{*}+1}}\left(\theta -\sigma_{r_{*}}\right){\left(\sigma_{z^{*}+1}-\sigma \right)}^{\omega -1}d\theta . \end{array} \end{array}$$

Now, we can deduce from (52) as follows by applying integration by substitution:

(53) $$\begin{array}{c} Y_{\omega ,r_{*},1}=h^{\omega +1}\frac{{\left(z^{*}+1-r_{*}\right)}^{\sigma }\left(z^{*}-r_{*}+2+\sigma \right)-{\left(z^{*}-r_{*}\right)}^{\sigma }\left(z^{*}-r_{*}+2+2\sigma \right)}{\omega \left(\omega +1\right)},\\ Y_{\omega ,r_{*},2}=h^{\omega +1}\frac{{\left(n+1-r_{*}\right)}^{\sigma +1}-{\left(z^{*}-r_{*}\right)}^{\sigma }\left(z^{*}-r_{*}+1+\sigma \right)}{\omega \left(\omega +1\right)}. \end{array}$$

Here, knowing *Y*_*ω*,*r*_∗_,1_ and *Y*_*ω*,*r*_∗_,2_, we simply substituted into (51) which then gives us the following numerical scheme:

(54) $$\begin{array}{c} \Theta \left(\sigma_{z^{*}+1}\right)=\Theta_{0}+\frac{1-\omega }{\nabla \left(\omega \right)}ℵ\left(\sigma_{z^{*}},\Theta \left(\sigma_{z^{*}}\right)\right)+\frac{\omega }{\nabla \left(\omega \right)}\times \overset{z^{*}}{\underset{r_{*}=0}{\sum }}\left[\frac{h^{\omega }ℵ\left(\sigma_{r_{*}},\Theta_{r_{*}}\right)}{\Gamma \left(\omega +2\right)}\left({\left(z^{*}+1-r_{*}\right)}^{\omega }\left(z^{*}-r_{*}+2+\omega \right)-{\left(z^{*}-r_{*}\right)}^{\omega }\left(z^{*}-r_{*}+2+2\omega \right)\right)\right]-\frac{\omega }{\nabla \left(\omega \right)}\overset{z^{*}}{\underset{r_{*}=0}{\sum }}\left[\frac{h^{\omega }ℵ\left(\sigma_{r_{*}-1},\Theta_{r_{*}-1}\right)}{\Gamma \left(\omega +2\right)}\left({\left(z^{*}+1-r_{*}\right)}^{\omega +1}-{\left(z^{*}-r_{*}\right)}^{\omega }\left(z^{*}-r_{*}+1+\omega \right)\right)\right]. \end{array}$$

Hence, we suggest the following fractional-order model for the Ebola-malaria coinfection model under the ABC-fractional derivative:

(55) $$\begin{array}{c} S_{H_{z^{*}+1}}=S_{H}\left(0\right)+\frac{1-\omega }{\nabla \left(\omega \right)}{ℵ}_{1}\left(\sigma_{z^{*}},S_{H}\left(\sigma_{z^{*}}\right)\right)+\frac{\omega }{\nabla \left(\omega \right)}\times \overset{z^{*}}{\underset{r_{*}=0}{\sum }}\left[\frac{h^{\omega }{ℵ}_{1}\left(\sigma_{r_{*}},S_{H_{r_{*}}}\right)}{\Gamma \left(\omega +2\right)}\left({\left(z^{*}+1-r_{*}\right)}^{\omega }\left(z^{*}-r_{*}+2+\omega \right)-{\left(z^{*}-r_{*}\right)}^{\omega }\left(z^{*}-r_{*}+2+2\omega \right)\right)\right]-\frac{\omega }{\nabla \left(\omega \right)}\overset{z^{*}}{\underset{r_{*}=0}{\sum }}\left[\frac{h^{\omega }{ℵ}_{1}\left(\sigma_{r_{*}-1},S_{H_{r_{*}-1}}\right)}{\Gamma \left(\omega +2\right)}\left({\left(z^{*}+1-r_{*}\right)}^{\omega +1}-{\left(z^{*}-r_{*}\right)}^{\omega }\left(z^{*}-r_{*}+1+\omega \right)\right)\right],\\ L_{E_{z^{*}+1}}=L_{E}\left(0\right)+\frac{1-\omega }{\nabla \left(\omega \right)}{ℵ}_{2}\left(\sigma_{z^{*}},L_{E}\left(\sigma_{z^{*}}\right)\right)+\frac{\omega }{\nabla \left(\omega \right)}\times \overset{z^{*}}{\underset{r_{*}=0}{\sum }}\left[\frac{h^{\omega }{ℵ}_{2}\left(\sigma_{r_{*}},L_{E_{r_{*}}}\right)}{\Gamma \left(\omega +2\right)}\left({\left(z^{*}+1-r_{*}\right)}^{\omega }\left(z^{*}-r_{*}+2+\omega \right)-{\left(z^{*}-r_{*}\right)}^{\omega }\left(z^{*}-r_{*}+2+2\omega \right)\right)\right]-\frac{\omega }{\nabla \left(\omega \right)}\overset{z^{*}}{\underset{r_{*}=0}{\sum }}\left[\frac{h^{\omega }{ℵ}_{2}\left(\sigma_{r_{*}-1},L_{E_{r_{*}-1}}\right)}{\Gamma \left(\omega +2\right)}\left({\left(z^{*}+1-r_{*}\right)}^{\omega +1}-{\left(z^{*}-r_{*}\right)}^{\omega }\left(z^{*}-r_{*}+1+\omega \right)\right)\right],\\ I_{U_{z^{*}+1}}=I_{U}\left(0\right)+\frac{1-\omega }{\nabla \left(\omega \right)}{ℵ}_{3}\left(\sigma_{z^{*}},I_{U}\left(\sigma_{z^{*}}\right)\right)+\frac{\omega }{\nabla \left(\omega \right)}\times \overset{z^{*}}{\underset{r_{*}=0}{\sum }}\left[\frac{h^{\omega }{ℵ}_{3}\left(\sigma_{r_{*}},I_{U_{r_{*}}}\right)}{\Gamma \left(\omega +2\right)}\left({\left(z^{*}+1-r_{*}\right)}^{\omega }\left(z^{*}-k+2+\omega \right)-{\left(z^{*}-r_{*}\right)}^{\omega }\left(z^{*}-r_{*}+2+2\omega \right)\right)\right]-\frac{\omega }{\nabla \left(\omega \right)}\overset{z^{*}}{\underset{r_{*}=0}{\sum }}\left[\frac{h^{\omega }{ℵ}_{3}\left(\sigma_{r_{*}-1},I_{U_{r_{*}-1}}\right)}{\Gamma \left(\omega +2\right)}\left({\left(z^{*}+1-r_{*}\right)}^{\omega +1}-{\left(z^{*}-r_{*}\right)}^{\omega }\left(z^{*}-r_{*}+1+\omega \right)\right)\right],\\ I_{D_{z^{*}+1}}=I_{D}\left(0\right)+\frac{1-\omega }{\nabla \left(\omega \right)}{ℵ}_{4}\left(\sigma_{z^{*}},I_{D}\left(\sigma_{z^{*}}\right)\right)+\frac{\omega }{\nabla \left(\omega \right)}\times \overset{z^{*}}{\underset{r_{*}=0}{\sum }}\left[\frac{h^{\omega }{ℵ}_{4}\left(\sigma_{r_{*}},I_{D_{r_{*}}}\right)}{\Gamma \left(\omega +2\right)}\left({\left(z^{*}+1-r_{*}\right)}^{\omega }\left(z^{*}-r_{*}+2+\omega \right)-{\left(z^{*}-r_{*}\right)}^{\omega }\left(z^{*}-r_{*}+2+2\omega \right)\right)\right]-\frac{\omega }{\nabla \left(\omega \right)}\overset{z^{*}}{\underset{r_{*}=0}{\sum }}\left[\frac{h^{\omega }{ℵ}_{4}\left(\sigma_{r_{*}-1},I_{D_{r_{*}-1}}\right)}{\Gamma \left(\omega +2\right)}\left({\left(z^{*}+1-r_{*}\right)}^{\omega +1}-{\left(z^{*}-r_{*}\right)}^{\omega }\left(z^{*}-r_{*}+1+\omega \right)\right)\right],\\ I_{T_{z^{*}+1}}=I_{T}\left(0\right)+\frac{1-\omega }{\nabla \left(\omega \right)}{ℵ}_{5}\left(\sigma_{z^{*}},I_{T}\left(\sigma_{z^{*}}\right)\right)+\frac{\omega }{\nabla \left(\omega \right)}\times \overset{z^{*}}{\underset{r_{*}=0}{\sum }}\left[\frac{h^{\omega }{ℵ}_{5}\left(\sigma_{r_{*}},I_{T_{r_{*}}}\right)}{\Gamma \left(\omega +2\right)}\left({\left(z^{*}+1-r_{*}\right)}^{\omega }\left(z^{*}-r_{*}+2+\omega \right)-{\left(z^{*}-r_{*}\right)}^{\omega }\left(z^{*}-r_{*}+2+2\omega \right)\right)\right]-\frac{\omega }{\nabla \left(\omega \right)}\overset{z^{*}}{\underset{r_{*}=0}{\sum }}\left[\frac{h^{\omega }{ℵ}_{5}\left(\sigma_{r_{*}-1},I_{T_{r_{*}-1}}\right)}{\Gamma \left(\omega +2\right)}\left({\left(z^{*}+1-r_{*}\right)}^{\omega +1}-{\left(z^{*}-r_{*}\right)}^{\omega }\left(z^{*}-r_{*}+1+\omega \right)\right)\right],\\ J_{z^{*}+1}=J\left(0\right)+\frac{1-\omega }{\nabla \left(\omega \right)}{ℵ}_{6}\left(\sigma_{z^{*}},J\left(\sigma_{z^{*}}\right)\right)+\frac{\omega }{\nabla \left(\omega \right)}\times \overset{z^{*}}{\underset{r_{*}=0}{\sum }}\left[\frac{h^{\omega }{ℵ}_{6}\left(\sigma_{r_{*}},J_{r_{*}}\right)}{\Gamma \left(\omega +2\right)}\left({\left(z^{*}+1-r_{*}\right)}^{\omega }\left(z^{*}-r_{*}+2+\omega \right)-{\left(z^{*}-r_{*}\right)}^{\omega }\left(z^{*}-r_{*}+2+2\omega \right)\right)\right]-\frac{\omega }{\nabla \left(\omega \right)}\overset{z^{*}}{\underset{r_{*}=0}{\sum }}\left[\frac{h^{\omega }{ℵ}_{6}\left(\sigma_{r_{*}-1},J_{r_{*}-1}\right)}{\Gamma \left(\omega +2\right)}\left({\left(z^{*}+1-r_{*}\right)}^{\omega +1}-{\left(z^{*}-r_{*}\right)}^{\omega }\left(z^{*}-r_{*}+1+\omega \right)\right)\right],\\ E_{M_{z^{*}+1}}=E_{M}\left(0\right)+\frac{1-\omega }{\nabla \left(\omega \right)}{ℵ}_{7}\left(\sigma_{z^{*}},E_{M}\left(\sigma_{z^{*}}\right)\right)+\frac{\omega }{\nabla \left(\omega \right)}\times \overset{z^{*}}{\underset{r_{*}=0}{\sum }}\left[\frac{h^{\omega }{ℵ}_{7}\left(\sigma_{r_{*}},E_{M_{r_{*}}}\right)}{\Gamma \left(\omega +2\right)}\left({\left(z^{*}+1-r_{*}\right)}^{\omega }\left(z^{*}-r_{*}+2+\omega \right)-{\left(z^{*}-r_{*}\right)}^{\omega }\left(z^{*}-r_{*}+2+2\omega \right)\right)\right]-\frac{\omega }{\nabla \left(\omega \right)}\overset{z^{*}}{\underset{r_{*}=0}{\sum }}\left[\frac{h^{\omega }{ℵ}_{7}\left(\sigma_{r_{*}-1},E_{M_{r_{*}-1}}\right)}{\Gamma \left(\omega +2\right)}\left({\left(z^{*}+1-r_{*}\right)}^{\omega +1}-{\left(z^{*}-r_{*}\right)}^{\omega }\left(z^{*}-r_{*}+1+\omega \right)\right)\right],\\ I_{M_{z^{*}+1}}=I_{M}\left(0\right)+\frac{1-\omega }{\nabla \left(\omega \right)}{ℵ}_{8}\left(\sigma_{z^{*}},I_{M}\left(\sigma_{z^{*}}\right)\right)+\frac{\omega }{\nabla \left(\omega \right)}\times \overset{z^{*}}{\underset{r_{*}=0}{\sum }}\left[\frac{h^{\omega }{ℵ}_{8}\left(\sigma_{r_{*}},I_{M_{r_{*}}}\right)}{\Gamma \left(\omega +2\right)}\left({\left(z^{*}+1-r_{*}\right)}^{\omega }\left(z^{*}-r_{*}+2+\omega \right)-{\left(z^{*}-r_{*}\right)}^{\omega }\left(z^{*}-r_{*}+2+2\omega \right)\right)\right]-\frac{\omega }{\nabla \left(\omega \right)}\overset{z^{*}}{\underset{r_{*}=0}{\sum }}\left[\frac{h^{\omega }{ℵ}_{8}\left(\sigma_{r_{*}-1},I_{M_{r_{*}-1}}\right)}{\Gamma \left(\omega +2\right)}\left({\left(z^{*}+1-r_{*}\right)}^{\omega +1}-{\left(z^{*}-r_{*}\right)}^{\omega }\left(z^{*}-r_{*}+1+\omega \right)\right)\right],\\ R_{M_{z^{*}+1}}=R_{M}\left(0\right)+\frac{1-\omega }{\nabla \left(\omega \right)}{ℵ}_{9}\left(\sigma_{z^{*}},R_{M}\left(\sigma_{z^{*}}\right)\right)+\frac{\omega }{\nabla \left(\omega \right)}\times \overset{z^{*}}{\underset{r_{*}=0}{\sum }}\left[\frac{h^{\omega }{ℵ}_{9}\left(\sigma_{r_{*}},R_{M_{r_{*}}}\right)}{\Gamma \left(\omega +2\right)}\left({\left(z^{*}+1-r_{*}\right)}^{\omega }\left(z^{*}-r_{*}+2+\omega \right)-{\left(z^{*}-r_{*}\right)}^{\omega }\left(z^{*}-r_{*}+2+2\omega \right)\right)\right]-\frac{\omega }{\nabla \left(\omega \right)}\overset{z^{*}}{\underset{r_{*}=0}{\sum }}\left[\frac{h^{\omega }{ℵ}_{9}\left(\sigma_{r_{*}-1},R_{M_{r_{*}-1}}\right)}{\Gamma \left(\omega +2\right)}\left({\left(z^{*}+1-r_{*}\right)}^{\omega +1}-{\left(z^{*}-r_{*}\right)}^{\omega }\left(z^{*}-r_{*}+1+\omega \right)\right)\right],\\ E_{EM_{z^{*}+1}}=E_{EM}\left(0\right)+\frac{1-\omega }{\nabla \left(\omega \right)}{ℵ}_{10}\left(\sigma_{z^{*}},E_{EM}\left(\sigma_{z^{*}}\right)\right)+\frac{\omega }{\nabla \left(\omega \right)}\times \overset{z^{*}}{\underset{r_{*}=0}{\sum }}\left[\frac{h^{\omega }{ℵ}_{10}\left(\sigma_{r_{*}},E_{EM_{r_{*}}}\right)}{\Gamma \left(\omega +2\right)}\left({\left(z^{*}+1-r_{*}\right)}^{\omega }\left(z^{*}-r_{*}+2+\omega \right)-{\left(z^{*}-r_{*}\right)}^{\omega }\left(z^{*}-r_{*}+2+2\omega \right)\right)\right]-\frac{\omega }{\nabla \left(\omega \right)}\overset{z^{*}}{\underset{r_{*}=0}{\sum }}\left[\frac{h^{\omega }{ℵ}_{10}\left(\sigma_{r_{*}-1},E_{EM_{r_{*}-1}}\right)}{\Gamma \left(\omega +2\right)}\left({\left(z^{*}+1-r_{*}\right)}^{\omega +1}-{\left(z^{*}-r_{*}\right)}^{\omega }\left(z^{*}-r_{*}+1+\omega \right)\right)\right],\\ I_{EM_{z^{*}+1}}=I_{EM}\left(0\right)+\frac{1-\omega }{\nabla \left(\omega \right)}{ℵ}_{11}\left(\sigma_{z^{*}},I_{EM}\left(\sigma_{z^{*}}\right)\right)+\frac{\omega }{\nabla \left(\omega \right)}\times \overset{z^{*}}{\underset{r_{*}=0}{\sum }}\left[\frac{h^{\omega }{ℵ}_{11}\left(\sigma_{r_{*}},I_{EM_{r_{*}}}\right)}{\Gamma \left(\omega +2\right)}\left({\left(z^{*}+1-r_{*}\right)}^{\omega }\left(z^{*}-r_{*}+2+\omega \right)-{\left(z^{*}-r_{*}\right)}^{\omega }\left(z^{*}-r_{*}+2+2\omega \right)\right)\right]-\frac{\omega }{\nabla \left(\omega \right)}\overset{z^{*}}{\underset{r_{*}=0}{\sum }}\left[\frac{h^{\omega }{ℵ}_{11}\left(\sigma_{r_{*}-1},I_{EM_{r_{*}-1}}\right)}{\Gamma \left(\omega +2\right)}\left({\left(z^{*}+1-r_{*}\right)}^{\omega +1}-{\left(z^{*}-r_{*}\right)}^{\omega }\left(z^{*}-r_{*}+1+\omega \right)\right)\right],\\ S_{V_{z^{*}+1}}=S_{V}\left(0\right)+\frac{1-\omega }{\nabla \left(\omega \right)}{ℵ}_{12}\left(\sigma_{z^{*}},S_{V}\left(\sigma_{z^{*}}\right)\right)+\frac{\omega }{\nabla \left(\omega \right)}\times \overset{z^{*}}{\underset{r_{*}=0}{\sum }}\left[\frac{h^{\omega }{ℵ}_{12}\left(\sigma_{r_{*}},S_{V_{r_{*}}}\right)}{\Gamma \left(\omega +2\right)}\left({\left(z^{*}+1-r_{*}\right)}^{\omega }\left(z^{*}-r_{*}+2+\omega \right)-{\left(z^{*}-r_{*}\right)}^{\omega }\left(z^{*}-r_{*}+2+2\omega \right)\right)\right]-\frac{\omega }{\nabla \left(\omega \right)}\overset{z^{*}}{\underset{r_{*}=0}{\sum }}\left[\frac{h^{\omega }{ℵ}_{12}\left(\sigma_{r_{*}-1},S_{V_{r_{*}-1}}\right)}{\Gamma \left(\omega +2\right)}\left({\left(z^{*}+1-r_{*}\right)}^{\omega +1}-{\left(z^{*}-r_{*}\right)}^{\omega }\left(z^{*}-r_{*}+1+\omega \right)\right)\right],\\ E_{V_{z^{*}+1}}=E_{V}\left(0\right)+\frac{1-\omega }{\nabla \left(\omega \right)}{ℵ}_{13}\left(\sigma_{z^{*}},E_{V}\left(\sigma_{n}\right)\right)+\frac{\omega }{\nabla \left(\omega \right)}\times \overset{z^{*}}{\underset{r_{*}=0}{\sum }}\left[\frac{h^{\omega }{ℵ}_{13}\left(\sigma_{r_{*}},E_{V_{r_{*}}}\right)}{\Gamma \left(\omega +2\right)}\left({\left(z^{*}+1-r_{*}\right)}^{\omega }\left(z^{*}-r_{*}+2+\omega \right)-{\left(z^{*}-r_{*}\right)}^{\omega }\left(z^{*}-r_{*}+2+2\omega \right)\right)\right]-\frac{\omega }{\nabla \left(\omega \right)}\overset{z^{*}}{\underset{r_{*}=0}{\sum }}\left[\frac{h^{\omega }{ℵ}_{13}\left(\sigma_{r_{*}-1},E_{V_{r_{*}-1}}\right)}{\Gamma \left(\omega +2\right)}\left({\left(z^{*}+1-r_{*}\right)}^{\omega +1}-{\left(z^{*}-r_{*}\right)}^{\omega }\left(z^{*}-r_{*}+1+\omega \right)\right)\right]\\ I_{V_{z^{*}+1}}=I_{V}\left(0\right)+\frac{1-\omega }{\nabla \left(\omega \right)}{ℵ}_{14}\left(\sigma_{z^{*}},I_{V}\left(\sigma_{z^{*}}\right)\right)+\frac{\omega }{\nabla \left(\omega \right)}\times \overset{z^{*}}{\underset{r_{*}=0}{\sum }}\left[\frac{h^{\omega }{ℵ}_{14}\left(\sigma_{r_{*}},I_{V_{r_{*}}}\right)}{\Gamma \left(\omega +2\right)}\left({\left(z^{*}+1-r_{*}\right)}^{\omega }\left(z^{*}-r_{*}+2+\omega \right)-{\left(z^{*}-r_{*}\right)}^{\omega }\left(z^{*}-r_{*}+2+2\omega \right)\right)\right]-\frac{\omega }{\nabla \left(\omega \right)}\overset{z^{*}}{\underset{r_{*}=0}{\sum }}\left[\frac{h^{\omega }{ℵ}_{14}\left(\sigma_{r_{*}-1},I_{V_{r_{*}-1}}\right)}{\Gamma \left(\omega +2\right)}\left({\left(z^{*}+1-r_{*}\right)}^{\omega +1}-{\left(z^{*}-r_{*}\right)}^{\omega }\left(z^{*}-r_{*}+1+\omega \right)\right)\right]. \end{array}$$

## 7. Numerical Results and Discussion

We illustrate the analytical results of this study by carrying out numerical simulations of the models using parameter values in Table 1 with initial values *S*_*H*_(0) = 1000, *L*_*E*_(0) = 270, *I*_*U*_(0) = 210, *I*_*D*_(0) = 300, *I*_*D*_(0) = 300, *I*_*T*_(0) = 320, *J*(0) = 200, *E*_*M*_(0) = 150, *I*_*M*_(0) = 800, *R*_*M*_(0) = 500, *E*_*EM*_(0) = 800, *I*_*EM*_(0) = 200, *S*_*V*_(0) = 650, *E*_*V*_(0) = 420, and *I*_*V*_(0) = 350. For the given sets of parameters in Table 1, we show the approximate solutions obtained using the considered iterative approaches against different fractional orders for each compartment, as seen in Figures 1–3. The illustrative graphs in Figures 1(a), 1(c), 1(d), 1(f), 2(b), 2(d), 2(e), 2(f), and 3(b) show no crossover effect but Figures 1(b), 1(e), 2(a), 2(c), and 3(a) show a crossover effect when the fractional order is changed.  Figure 4 shows the fractional dynamics when one varies the malaria treatment rate with a fractional order of *σ* = 0.90. It shows that an increasing treatment rate reduces the number of infected individuals with malaria but does not affect the number of infected individuals with Ebola.  Figure 5 shows the dynamics of the disease when one increases the rate of treatment of individuals infected with Ebola.  Figure 6 shows the fractional dynamics when one varies the Ebola detection rate with a fractional order of 0.9. In a nutshell, we notice that the variation in the treatment rate for malaria does not affect susceptible individuals. *S*_*H*_, individuals that are latently infected with the Ebola virus *L*_*E*_(*t*), Ebola virus afflicted people who went unnoticed *I*_*U*_, individuals who have been infected with the Ebola virus and have been diagnosed with the disease *I*_*D*_, persons undergoing Ebola virus therapy *I*_*T*_, isolated Ebola individuals *J*, malaria-exposed population *E*_*M*_, individuals who are infected with the Ebola virus and at the risk of contracting malaria *E*_*EM*_, persons infected with Ebola and malaria *I*_*EM*_, and the vector population *N*_*V*_ = *S*_*V*_ + *E*_*V*_ + *I*_*V*_. Similarly, when one varies the treatment rate for Ebola, we notice that the following compartment is not affected; thus, susceptible individuals *S*_*H*_, Ebola virus afflicted people who went unnoticed *I*_*U*_, malaria-exposed population *E*_*M*_, individuals who are infected with the Ebola virus and at the risk of contracting malaria *E*_*EM*_, individuals infected with Ebola and malaria *I*_*EM*_, individuals affected with malaria only *I*_*M*_, recovered individuals from malaria *R*_*M*_ and the vector population *N*_*V*_ = *S*_*V*_ + *E*_*V*_ + *I*_*V*_. The graphical dynamics of the variation in the detection rate indicate that the variation in the detection rate only affects the following compartments: individuals that are latently infected with the Ebola virus *L*_*E*_(*t*), Ebola virus afflicted people who went unnoticed *I*_*U*_, individuals who have been infected with the Ebola virus and have been diagnosed with the disease *I*_*D*_, and people undergoing Ebola virus therapy *I*_*T*_.

## 8. Conclusion

This paper considers Ebola-malaria coinfection under the Mittag-Leffler kernel fractional derivative. We have determined epidemiological, computational, and theoretical inferences to understand better how to prevent the Ebola, malaria, and Ebola-malaria coinfections simultaneously in the human population. In a prior mathematical investigation into Ebola-malaria coinfections, the fractional derivative was not taken into account. As a result, our research adds up to the dynamic analysis of Ebola, malaria, and Ebola-malaria coinfections. First and foremost, we guaranteed solutions' existence and uniqueness by using the Krasnoselskii's type and the Banach fixed point theorem. HU stability ensured the model's stability. The simulation has been given with the help of the Lagrange interpolation to solve the considered problem analytically. Our results reveal that the prevalence of the Ebola, malaria and Ebola-malaria coinfections varied from low to moderate depending on the fractional operators. In addition, we observed from our solutions that there was no significant difference in the Ebola-malaria coinfections of the immune response. Moreover, Ebola-malaria coinfection-related mortality varied from moderate to high depending on the fractional operators. Hence, we conclude that the global nature of ABC-fractional order dynamics excellently explains the coinfection model characteristics. Thus, the concept in this paper has crucial implications for biological models and their problems, and it is helpful for Ebola-malaria coinfection analysis and control strategy. In future work, different fractional order derivatives and their theoretical and numerical stability can be investigated with other control measures.

## Figures and Tables

**Figure 1:** Fractional dynamics of different classes at different fractional order *σ*.

**Figure 2:** Fractional dynamics of different classes at different fractional order *σ*.

**Figure 3:** Fractional dynamics of different classes at different fractional order *σ*.

**Figure 4:** Fractional dynamics when one varies malaria treatment rate with fractional order *σ* = 0.90.

**Figure 5:** Fractional dynamics when one varies Ebola treatment rate with fractional order *σ* = 0.90.

**Figure 6:** Fractional dynamics when one varies Ebola detection rate with fractional order *σ* = 0.90.

**Table 1:** Parameter values in the model.

Parameters	Values	Sources	Parameters	Values	Sources
*π*_*H*_	800	Assumed	*r*, *γ*_*UE*_	0.05, 0.003	Assumed
*π*_*V*_	500	Assumed	*θ*	0.028	Assumed
*μ*	1/65 × 365	Forecasted	*η*_*EM*_	0.08	Assumed
*τ*_1_	0.009	Assumed	*η*_*D*_	0.01	Assumed
*τ*_3_	0.013	Assumed	*ρ*	0.0095	Assumed
*ε*_1_, *ε*_2_	0.0001, 0.001	Assumed	*σ*_1_, *σ*_2_	0.001, 0.001	[16]
*δ*_*IM*_	0.003	Assumed	*b*	0.0031	Assumed
*K*_*E*_	0.0008	Assumed	*β*_*V*_	0.008	Assumed
*δ*_*UE*_, *δ*_*DE*_	0.0027, 0.008	[17, 18]	*ϕ*_1_	0.018	Assumed
*σ*_*V*_	0.1	[17]	*ϕ*_3_	0.0012	[16]
*β*_*E*_, *β*_*EM*_	0.080, 0.080	Assumed	*K*_*M*_, *K*_*EM*_	0.008, 0.008	Assumed
*η*_1_, *η*_2_	0.034, 0.067	Assumed	*δ*_*j*_, *δ*_*EM*_, *δ*_*IEM*_	0.008, 0.003,0.008	Assumed
*β*_*M*_	0.04	Assumed	*ε*_3_	0.082	Assumed
*ϕ*_2_	0.028	Assumed	*τ*_4_	0.0069	[18]
*ω*_1_	0.021	Assumed	*τ*_2_	0.0018	Assumed
*η*_*T*_	0.0018	Assumed	*μ*_*V*_	0.004	Assumed
*η*_*J*_	0.01	Assume			

## Data Availability

No data is used for this study.
